# Intelligent Scanning Detection System of Muscle Exercise Fatigue Based on Surface Electromyography

This article has been retracted.

**DOI:** 10.1155/2022/9163978

**Published:** 2022-08-27

**Authors:** Weiqi Wang

**Affiliations:** Fuyang Normal University, Fuyang, Anhui 236037, China

## Abstract

In order to use the surface EMG signal to *automatically* detect the muscle fatigue state, a research method of the muscle exercise fatigue intelligent scanning detection system based on surface EMG was proposed, and the sEMG signal features of 10 subjects before and after fatigue were extracted. A time-varying parameter autoregressive model is established. By introducing the Legendre basis function, the parameter identification of the linear nonstationary process is transformed into the parameter identification of the linear time-invariant system. Combined with the correlation index, the optimal Legendre base function dimension of the time-varying system parameter estimation can be obtained, then the best model fitting effect can be obtained, and the time-invariant parameters are solved by the least square method. Using the rate of change of the first time-varying parameter (ARC1) of the autoregressive model before and after fatigue as an index to detect muscle fatigue sensitivity, a two-tailed *t* test was used to compare the mean power frequency (MPF) and the median frequency (MF) with the rate of change. The results showed that the change rates of ARC1, MPF, and MF before and after fatigue were34.33% ± 2.5%, 68% + 2.03%, and 22.80% + 2.19%, which were 41% and 25%, respectively. The rate of change of ACR1 was significantly higher than that of MPF and MF (*P* < 0.05). When detecting muscle fatigue by sEMG signal, it has the advantages of short time and high sensitivity. It can be used for online real-time analysis of muscle fatigue, providing a potential analysis tool for limb muscle strain, rehabilitation, and ergonomics assessment.

## 1. Introduction

Exercise-induced muscle fatigue refers to the physiological phenomenon that exercise causes the muscle to produce the maximum random contraction force or the temporary decline of output power [1]. Its mechanism is extremely complex, involving a variety of physiological processes, such as central motor drive, neuromuscular junction excitation contraction coupling, and muscle energy metabolism. In recent years, with the development of electromyography technology, using EMG to record and study muscle fatigue has become a more and more common method in physiology, as shown in Figure 1. EMG technology has the advantages of noninvasive, real-time, and multitarget measurement [2]. The study of EMG can reveal the mechanism of muscle fatigue, for example, to judge fatigue in sports practice and guide training. It is especially suitable for measuring changes in EMG during exercise, and EMG will gradually be used in many aspects of sports science research. The analysis of EMG signal mainly includes time domain and frequency domain analysis. The time domain analysis of EMG can provide us with the discharge time, total discharge amount, discharge frequency, and discharge amplitude of various muscle fibers under the electrode, especially in the analysis of movement technology. The EMG frequency domain analysis can provide us with the following information: we can know the concentration trend of discharge energy at a certain frequency, the mobilization of different types of muscle fibers, and the relationship between the change of neuromuscular function and the change of discharge frequency. For clarifying the working mechanism and functional state of nerve and muscle, the best way is to apply time domain and frequency domain analysis at the same time, especially the latter. In the static working state, the more consistent conclusion is that the amplitude value of iEMG from initial state to fatigue state increases with the deepening of fatigue degree, and the power spectrum of frequency domain value shifts to low frequency. In addition, the specific range of frequency reduction was clearly obtained. They concluded that the left shift value of the corresponding frequency of the maximum spectral peak was (9-18 Hz). In addition to the change in the recruitment form of fast and slow muscle fiber components during skeletal muscle contraction, i5s may also be caused by the hyperpolarization of muscle cell membrane potential caused by the increase of pH value in muscle tissue, resulting in the outflow of K+ in cells. K+ outflow will block the hyperpolarization of cell membrane potential and reduce the excitability of muscle cells and the conduction velocity of muscle fibers, resulting in the transfer of muscle discharge frequency to low frequency band [3]. However, we do not rule out this possibility: according to the current research, muscle tissue has the function of low-pass filtering. During muscle contraction, the length of the muscle is shortened, the thickness is increased, and the distance between the recording electrode and the moving unit is increased, resulting in the filtering of some high-frequency signals and the increase of the proportion of low-frequency signals and resulting in the low shift of the spectrum.

## 2. Literature Review

Er and Erk found that muscle activity is a complex exercise under the control of the central nervous system. Muscle fatigue usually refers to the temporary decline of the maximum work capacity or maximum contraction capacity of the system [4]. Fan and others have shown that there have been different opinions on the mechanism of exercise-induced muscle fatigue for a long time [5]. In fact, Ben et al. have found that the human body is a complex organism, and various systems and organs are not isolated, but interconnected and restricted under the regulation of the nervous system [6]. The essence of fatigue is the weakening of the function of the transverse bridge of muscle fibers and matrix network, resulting in the weakening of muscle filament sliding. Shaoting and others found that ADP/ATP increased in the triple tube structure, resulting in the decrease of calcium uptake by the matrix network. The surface EMG signal is the bioelectric signal recorded during the activity of the neuromuscular system guided by the electrode from the skin surface. It has different degrees of correlation with the activity state and function of the muscle, so it can reflect the activity of the neuromuscular system to a certain extent [7]. Lindinger and Cairns found that electromyography measurement generally uses three electrodes, two electrodes are placed at the part where the action potential can be measured and amplified, and the third electrode is the grounding electrode. Before placing the electrode, the body hair of the measurement part should be scraped off, the skin should be cleaned with fine sand and absolute ethanol, and conductive paste should be used to reduce the impact of skin resistance on electromyography signal [8]. Most scholars believe that the position of the surface electrode should be as close to the abdominal center as possible to obtain the maximum EMG signal from the rhomboid muscle. Dong and others believe that by sticking the electrode to the geometric center of muscle contraction and the electrode direction along the longitudinal axis of muscle fiber, the measured EMG signal is the most reliable, the two electrodes gather for 2-3 cm, and the ground wire is connected to a relatively stable place when moving close to the electrode, so the collected EMG signal is the most stable [9]. Greco and others found that the surface electrode can comprehensively reflect the activity of this part of the muscle. Surface electromyography collects one-dimensional time series signals [10]. It is the superposition of electrode changes in time and space when the surface guide electrode touches multiple moving units. From a physiological point of view, Tang and others are related to the fiber composition and anatomical structure of muscle, the number of motor units participating in activities under different functional and active states, the discharge frequency of different motor units, the degree of synchronization of motor unit activities, and the recruitment mode of motor units [11]. The influence of adipose tissue on the test results is greater when muscle is relaxed than when muscle is moving, but it does not affect the symmetry of both sides. EMG signals can be derived from random contraction and electrical induction. Random contraction EMG signals are the sum of action potentials of many motor units. During electrical induction, Sunayana and others found that due to external stimulation, motor unit action potential synchronization produced an exact evoked response, namely, M wave. This recording method can help us confirm the most superficial motor unit, which is more rapid than muscle fatigue caused by random contraction, and the obtained EMG signal has less change and more stable [12]. Grabowski and others found that in recent years, with the rapid development of computer, the quantitative analysis of electromyography has become possible. SEMG signal analysis includes time domain analysis and frequency domain analysis [13]. Kou and Zhang believe that its detection has the advantages of noninvasive, real-time, and multitarget measurement [14]. SEMG signal analysis is a means and method to find the change law and characteristics of sEMG signal by using the theory and method of signal analysis. Time domain analysis can provide us with the discharge time, total discharge amount, discharge frequency, discharge amplitude, etc. of muscle fibers, especially in the motion analysis of sports technology. Frequency domain analysis can provide us with the following information: The mobilization of different types of muscle fibers, the energy supply state of neuromuscles, and the concentration trend of discharge are at a certain frequency. For practical application, time domain and frequency domain analysis should be used at the same time.

## 3. Method

The subjects were 10 healthy men, who had no history of upper limb muscle strain, normal body mass index, and did not participate in any violent activities within 24 hours before the experiment. Before the experiment, each subject received the experiment notice, signed the informed consent, and conducted the experiment action training. The experiment was conducted in a key laboratory of medical engineering. Before the experiment, the laboratory adjusted the temperature to 279°C, removed the jewelry of the subject, and put the electrode piece in the middle of the biceps brachii of the right upper limb. The right hand of each group of subjects is upward, the upper arm is parallel to the body, and the angle between the forearm and the upper arm elbow is 90°. Hold 1.5 kg dumbbell and start isometric contraction until the subjects subjectively feel that muscle fatigue cannot continue. Collect and record the data of the early and late stage of biceps brachii fatigue of the right upper limb. Due to the large differences in age and individual among each subject, it is required that the dumbbell weight and electrode placement position must be consistent [15]. Experimental equipment and materials: before the experiment, prepare the experimental equipment and materials, including computer, wireless surface EMG acquisition system (including 1 DTS EMG sensor, 1 DTS desktop receiving box, 1 double electrode clamp, 5 V DC charging line, mini USB data line, and 1 elastic fixing belt), 2 electrode pieces, alcohol, cotton swab, and subject information. The brand is Noraxon, the model is sEMG sensor signal acquisition system, and the version is mr3 6 software. The wireless surface electromyography signal sensor is used. The disposable Ag/AgCl electrode sheet is used. The time constant is set to 0.05 s, and the sampling frequency is 1500 Hz. The disposable electrode sheet is pasted according to the muscle model, and the spacing between the electrode sheets is 20 mm. Because the sEMG signal is relatively weak, the useful signal is distributed in the frequency range of 0 ~500 Hz, and the main energy part is distributed in the frequency range of 50~150 Hz. Surface EMG signals detected by body surface electrodes mainly include power frequency interference (50 Hz), baseline drift, and ECG interference (5 ~ 20 Hz). These noises will seriously affect the quality of surface EMG signals [16]. In order to enhance the effective components of sEMG signal and suppress noise and artifacts, the effective elimination of noise is very important for the subsequent processing of sEMG signal. Butterworth 20~500 Hz band-pass filter is used to eliminate baseline drift and ECG interference, and Butterworth band stop filter is used to eliminate 50 Hz power frequency interference. There are differences in muscle activity among different subjects. In order to uniformly compare the effects of different parameter eigenvalues on fatigue characterization, it is necessary to normalize the surface EMG signal [17].

In this experiment, the autoregressive model (AR) describes a “short-term stable” random process. The observed value *x*_*n*_ of the random process at this time is correlated with the observed value *x*_*n*−1_ before that time. The calculation formula of autoregressive model with p-order parameters is shown in the following formula:

(1) $$\begin{array}{c} x_{n}=-\overset{p}{\underset{i=1}{\sum }}a_{i}\left(n\right)x_{n-i}+e_{n}, \end{array}$$

where *a*_*i*_(*n*) is the autoregressive coefficient and also the parameter of AR (*P*) model; *n* = 1, 2, ⋯, *N*, *N* is the length of sampling data; *e*_*n*_ is a stationary white noise process; *x*_*n*_ is the observation value, and *x*_*n*−*i*_ is the observation sequence value.

Since the sampling frequency of the EMG acquisition equipment is 1500 Hz, the time-varying system parameters change too fast, and the convergence of the adaptive algorithm is defective. Therefore, the basis function expansion method is used [18]. The basis function expansion method is used to identify the time-varying system. Is the time-varying coefficient *a*_*i*_(*n*) expressed as a linear combination of a set of basis functions? See the following equation:

(2) $$\begin{array}{c} ai\left(n\right)=\overset{m}{\underset{j=1}{\sum }}a_{ij}\left(n\right)f_{i}\left(n\right), \end{array}$$

where *a*_*i*_*j*__ is the time invariant coefficient of the expansion, *f*_*j*_(*n*) is the basis function, and *M* is the extended dimension of the basis function.

Then, equation (2) can be rewritten as

(3) $$\begin{array}{c} X=BA+e. \end{array}$$

Using the basis function expansion, the identification problem of *P* time-varying coefficients in the time-varying model formula (1) is transformed into the identification of *P* × *M* constant parameters, that is, the parameter identification of the original nonstationary process is transformed into the identification of a linear time invariant system [19]. After the model is expressed in matrix form, the estimated value $\overset{\wedge }{A}$ of time invariant parameter *a* is solved by the least square method, as shown in the following formula:

(4) $$\begin{array}{c} \overset{\wedge }{A}={\left(B^{T}B\right)}^{-1}B^{T}+e. \end{array}$$

Substitute equation (4) into equation (2) to obtain the estimated value $\overset{\wedge }{a_{i}}\left(n\right)$ of time-varying parameter *a*_*i*_(*n*).

Frequency domain analysis is to analyze the characteristics of sEMG signal from the perspective of frequency. The method is to obtain the spectrum or power spectrum of sEMG signal after short-time Fourier transform. The common analysis parameters of frequency domain analysis are MPF and MF. Because MPF and MF are based on short-time Fourier analysis, their time and resolution are fixed. However, for surface myoelectric signals, when the spectrum distribution range is wide, it is difficult to find a suitable time window for analysis, that is, their time and frequency resolution are low.

By comparing and analyzing the change rate (CR) of the fatigue index before and after fatigue of the three methods, we can determine which characteristic parameter value index has higher sensitivity to muscle fatigue response, and further explain which method is suitable to characterize muscle fatigue. The change rate of relevant characteristic parameter values before and after fatigue is defined in the following formula:

(5) $$\begin{array}{c} \text{CR}=\frac{\left({\text{y}}_{i+M}-{\text{y}}_{i}\right)}{y_{i}\times 100\%}, \end{array}$$

where*y* and*y*_*i*_ are the value before fatigue, and *y*_*i*+*m*_ is the value after fatigue.

After calculation, the MPF of surface EMG signals before and after fatigue is 208.34 and 149.35 Hz, respectively, and the MF is 132.98 and 104.75 Hz, respectively. The MPF change rate obtained from equation (5) is -28.68%, and the MF change rate is -21.66%. Because MPF and MF are based on the principle of short-time Fourier, they have long sampling time, poor real-time performance and resolution. In order to compare the sensitivity of the three methods to muscle fatigue, the following MPF and MF eigenvalues are calculated based on the data length of *n* = 15000 points (*t* = 10 s). Based on the characteristics of time-varying AR model, such as short sampling time and rapid response to time, the corresponding time-varying parameters can be obtained by using time-varying parameter AR model to process the first *n* = 150 point (*t* = 0.1 s) data before and after fatigue. After calculation, the ARC1 of surface EMG signals before and after fatigue is -2.35 and -3.79, respectively. The change rate of ARC1 obtained from equation (5) is 37.39%. The time-varying autoregressive model method analyzes the surface EMG signal from the perspective of least mean square error fitting, which overcomes the shortcomings of low frequency resolution and poor variance performance of classical spectrum estimation. Compared with the short-time Fourier transform analysis, it overcomes the problem that the sampling time of sEMG signal is long enough for the traditional extraction of frequency-domain parameters. Taking the sampling frequency of 1500 Hz and 512 points of time window as an example, the shortest data also needs 512/1500 ≈ 0.34 s > 0.1 s when calculating MPF and MF parameters.

The data analysis module of Excel 2013 software is adopted. The two tailed *t*-test analysis method is used to analyze the statistical difference of the sensitivity effect of each parameter eigenvalue on fatigue response, that is, to analyze the statistical difference of each parameter eigenvalue on the characterization effect of muscle fatigue degree. Statistical steps of change rate data: *F* test shall be conducted first, which is also called variance homogeneity test. *F*-test is used in the two sample *t*-test. The purpose of *F*-test is to determine whether to use the two sample equal variance *t*-test or the two sample heteroscedasticity *t*-test. If the two times of one tailed *P* value of *F* test is greater than 0.05, it indicates that there is no significant difference between the two variances, then double sample equal variance *t* test is used. Otherwise, a two sample heteroscedasticity *t*-test is selected.

## 4. Experiment and Discussion

Figure 2 shows the surface EMG signal diagram of biceps brachii of a typical subject. It can be seen that the amplitude of surface EMG signal of muscle before and after fatigue tends to increase, which reflects the increase in the number of exercise units participating in activities from muscle contraction to fatigue, which is reflected in the increase in the amplitude of surface EMG signal during muscle fatigue [20].

Figure 3 shows that the correlation index l obtained by estimating the 6th order AR model based on the basis function expansion method of a typical subject changes with the dimension of the basis function, and the optimal dimension of Legendre basis function is obtained from equation (10) [21]. As can be seen from Figure 3, when the dimension of the basis function *m* ≥ 4, the parameter identification effect fluctuates little and tends to be stable. A large number of experiments show that the parameter identification effect is the best when *P* = 6 and *M* = 7.

Figure 4 shows the time-varying parameter identification results of a typical subject based on Legendre expansion method. It can be seen that the Legendre expansion method can better track the signal because of its good local characteristics, and the identification result is relatively smooth, especially there is no sudden change of parameter position at the peak and trough [22]. Therefore, Legendre expansion method has ideal identification effect.

Table 1 shows the fatigue characteristic values of subjects before and after fatigue. The experimental results show that 10 groups of time-varying parameters are obtained. The first parameter of each group of AR model (ARC1) is the most important. It directly reflects the relationship between the current time and the previous time. It is the most direct quantity of the change of muscle state with time. Each order of AR parameters changes with time point. ARC1 in the estimated signal 0.1 s time period is calculated as the index to evaluate muscle fatigue state. MPPF and MF within 10 s of the estimated signal are calculated as indicators for evaluating muscle fatigue [23].

From the change trend of characteristic parameters before and after fatigue, ARC1, MPF, and MF show a decreasing trend. From the change rate of characteristic parameters before and after fatigue, the change rate of ARC1 is high. AR model is adopted to overcome the problem that MF and MPF require long enough sampling time of sEMG signal [24]. The change rates of MPF, MF, and ARC1 of 10 subjects before and after fatigue were taken as fatigue indicators. The change rates were statistically analyzed. The mean value and standard deviation of the change rates were 25.68% + 2.03%, 22.80% + 2.19%, and 34.33% + 2.41%, respectively. Because there are significant differences between ARC1 and MPF and between ARC1 and MF, which are significantly higher than MPF and MF, respectively, it shows that using ARC1 parameter index to track muscle fatigue has high resolution sensitivity [25].

Legendre basis function is used to expand the parameters of linear time-varying system under white noise excitation, and the correlation index is used to select the best dimension of Legendre basis function. Through the experimental study of muscle fatigue, the characteristic parameters analyze the characterization effect of muscle fatigue. Through experiments, ARC1 is compared with traditional frequency domain parameters MPF and MF to prove the feasibility and effectiveness of ARC1 in the field of evaluating muscle fatigue [26].

## 5. Conclusion

The Legendre basis function expansion method is used to transform the identification problem of linear nonstationary process into the identification problem of linear time invariant system. The surface EMG signals of 10 subjects were extracted. The change rate of ARC1 in a short time was used as the index to evaluate the sensitivity of muscle fatigue. The experiment proved that it was more sensitive to fatigue response than MPF and MF, so it had the effect of amplifying the subtle feature information and making the unobvious feature information obvious.

The detection of muscle fatigue by sEMG signal can not only better characterize the change degree of muscle fatigue but also has the advantages of short time and high sensitivity. It can be applied to online and real-time detection of muscle fatigue and provide a reliable analysis tool for upper limb muscle strain assessment, rehabilitation treatment, and ergonomics research. The problem of time-varying parameter identification has always been a research difficulty in academic circles. It can be seen from the fact that the sensitivity of ARC1 in 10 subjects is higher than that of MPF and MF. This research method has applicability. In order to further verify and consolidate the correctness and practicability of the above results, in addition to a large number of simulations to verify that the experiment has the advantages of short time and high sensitivity, a large number of experiments still need to be carried out in the later stage of the next research, so as to further improve its practical value in the fields of muscle fatigue judgment.

## Figures and Tables

**Figure 1:** Detection of muscle exercise fatigue.

**Figure 2:** (a) Surface electromyography prefatigue. (b) Surface electromyography late fatigue.

**Figure 3:** (a) Correlation index changes with the dimension of basis function before fatigue. (b) Correlation index changes with the dimension of basis function after fatigue.

**Figure 4:** (a) Time-varying parameter identification results based on Legendre expansion method before fatigue. (b) Time varying parameter identification results based on Legendre expansion method after fatigue.

**Table 1:** Fatigue characteristic value and its change rate of each subject (before and after fatigue).

Subject	Average power frequency/MPF			First parameter of AR model/ARCI			Median frequency/MF		
	Before fatigue/Hz	After fatigue/Hz	Change rate/%	Before fatigue	After fatigue	Change rate/%	Before fatigue/Hz	After fatigue/Hz	Change rate/%
1	209.33	149.30	26.86	-2.25	-3.09	37.39	132.95	104.15	21.66
2	171.83	128.63	25.21	-2.12	-2.75	34.95	123.19	96.28	21.85
3	199.56	143.22	25.14	-2.41	-3.17	29.77	126.82	100.48	20.77
4	161.30	125.44	28.23	-1.89	-2.50	31.74	122.61	90.69	26.03
5	190.10	137.63	22.23	-2.18	-2.92	32.18	128.78	101.28	21.36
6	193.21	148.57	27.60	-2.42	-3.30	33.92	145.59	109.47	24.81
7	148.49	112.36	23.10	-2.26	-3.05	36.14	96.09	76.74	20.13
8	190.69	137.96	24.33	-2.72	-3.44	35.12	126.38	99.26	21.46
9	174.80	130.73	27.65	-2.00	-2.71	36.47	128.08	97.38	23.97
10	207.28	152.47	26.44	-2.09	-2.84	35.66	165.79	122.76	25.95
Mean ± SD	25.68 ± 2.03			34.33 ± 2.41			22.80 ± 2.19		

## Data Availability

The data used to support the findings of this study are available from the corresponding author upon request.
